# “Moving on to an Open World”: A Study of Participants' Experience in Meaningful Activities and Recovery (MA&R)

**DOI:** 10.1155/2022/7418667

**Published:** 2022-11-08

**Authors:** Nanna Kaas Tepavicharov, Jeanette Reffstrup Christensen, Tom Møller, Lene Falgaard Eplov, Siv Therese Bogevik Bjørkedal

**Affiliations:** ^1^Research Unit for General Practice, Department of Public Health, University of Southern Denmark, J.B. Winsløws Vej 9A, DK-5000 Odense C, Denmark; ^2^Research Unit for General Practice & Research Unit for User Perspectives and Community-Based Intervention, Department of Public Health, University of Southern Denmark, J.B. Winsløws Vej 9A, DK-5000 Odense C, Denmark; ^3^Research Unit for General Practice, Bartholins Allé 2, 8000 Aarhus, Denmark; ^4^CKO University Hospital of Copenhagen Rigshospitalet Dep. 8513, 2100 Copenhagen, East, Denmark; ^5^University of Copenhagen, Denmark; ^6^CORE: Copenhagen Research Center for Mental Health, Team for Inclusion and Recovery, Gentofte Hospitalsvej 15, Opg. 3A, 2900 Hellerup, Denmark

## Abstract

**Background:**

Meaningful activities and Recovery (MA&R) is a peer coled occupational therapy intervention, to support occupational engagement among persons with psychiatric disabilities.

**Aim:**

To investigate participants' perspectives on how MA&R influenced occupational engagement and recovery processes. *Material and Methods*. A qualitative study with a phenomenological-hermeneutic design. Individual semistructured interviews were conducted with three women and ten men who had participated in MA&R. Participants were recruited from community mental health centres and municipality mental health services in two Danish municipalities. Analysis strategy was based on Malterud's Systematic Text Condensation.

**Results:**

MA&R was perceived as a practical approach to recovery, by providing an opportunity for reorientation, meaning, making in mundane activities, and a new outlook on everyday life. Participating in MA&R challenged a black and white approach to activities, put emphasis on “the little things”, and enhanced curiosity, presence, and joy in occupational engagement.

**Conclusion:**

MA&R supported participants in developing a new “lens” on meaningful activities. The lens enhanced occupational engagement and made it possible to live according to personal preference. Results can inform further development and delivery of recovery-oriented occupational therapy interventions and add to the understandings of how occupational engagement and recovery are intertwined and manifested through everyday experiences. Thus, occupational engagement is an important target for recovery-oriented interventions. Occupational therapists and peer-workers coleading such interventions is feasible and makes good sense to the participants.

## 1. Introduction

Mental disorders are one of today's largest public health challenges, estimated to affect 38 percent of the EU population each year [1, 2]. Mental illnesses impact peoples' functioning and quality of life [3–7], as well as their abilities and opportunities for occupational engagement [8–10]. Research has found that what people do, such as time spent in a variety of activities and how they feel about what they do in terms of valued and satisfied activities, are important for health and well-being [9, 11–14]. Occupational engagement has been described by Black et al. [15] as; the active involvement in occupation, finding value and meaning, balanced engagement, subjective experience of engagement, developing identity through occupation, and social and environmental interactions. Occupational engagement plays a significant part in the recovery process [16–18]. Personal recovery is a unique and personal experience that encompasses hope, identity, meaning, and personal responsibility [19–21]. Regardless of the presence of mental illness, recovery is an ongoing process and a journey of finding ways to a meaningful life and developing valued social roles in the community, working towards better mental health [22–24]. Five key components for personal recovery process' have been identified under the acronym CHIME Connectedness, Hope and optimism, Identity, Meaning and purpose in life, and Empowerment [20].

Research investigating the links between recovery and occupational engagement has found that recovery is experienced through engagement in ordinary everyday activities in line with the “normal” roles and responsibilities, hereby rebuilding hope and connecting to an ordinary life in the community. [16, 17, 25–28]. Although a link between occupational engagement, well-being, and recovery has been established, there are only few evidence-based interventions targeting engagement in activities. More knowledge is therefore needed on how engagement in meaningful activities can be supported as a crucial part of the recovery process [29–31]. To address this, manualized programs [32–34] have been developed and investigated, to inform occupational therapists in mental health and how they can help patients support occupational engagement. Among the programs are Balancing Everyday Life (BEL) [32, 35–37], Action Over Inertia (AOI) [33, 38, 39], and the Occupation Matters Programme (OMP) [34] Occupation Matters and Balancing Everyday Life (BEL) are explicitly informed by previous lifestyle interventions such as the Lifestyle Redesign approach whereas the Action Over Inertia (AOI) manually describes its conceptual foundations as rooted in CMOP-E, recovery, Do-Live-Well, and capabilities frameworks. [14, 32–34] The programs provide knowledge on, and stimulate to reflections about occupations in relation to health, wellbeing, and recovery [32–34]. BEL and AOI both revolve around reengagement in healthy, satisfying, and varied occupational patterns (occupational balance) [32, 33], while OPM focuses on reengaging in occupations and redesigning lifestyle that facilitate recovery [34]. The interventions are led by occupational therapists, have a group-based format (AOI can also be delivered as a one-on-one intervention), and utilize various strategies such as home assignments and peer-support among group participants to facilitate change processes in relation to occupational patterns and occupational engagement [32, 34, 35, 37, 38]. Qualitative studies with participants with mental illness have found that reengaging in occupations during recovery often is a hard and demanding process [38, 40, 41]. It has been suggested that advancing occupational therapy interventions by offering individual support and incorporating collaborations between occupational therapists and peer-workers, may hold unrealized potentials for supporting occupational engagement and recovery [38, 40, 42]. Peer-workers are people with personal experiences with mental health problems, employed in mental health services to explicitly use their experiences to support others in their recovery [43].

Meaningful Activities and Recovery (MA&R) is a novel curriculum-based program to facilitate occupational engagement among persons with psychiatric disabilities [44]. MA&R differs from the earlier-described interventions, by (i) combining group sessions with one-on-one meetings (taking place interchangeably), (ii) being coled by a peer-worker and an occupational therapist, (iii) offering participants individual support to explore, engage, and practice occupational engagement in their homes or community, and (iv) have a longer duration in time. MA&R lasts for approximately eight months, whereas BEL, OMP, and AOI last between two to five months [44]. MA&R was investigated in a randomized controlled trial (RCT) for its effectiveness. However, the RCT design does not allow gaining insights into how MA&R was perceived by the participants, or how they experienced changes in occupational engagement and recovery during the intervention. The rationale for conducting this study was therefore, to provide a better and more nuanced understanding of the change processes in relation to occupational engagement and recovery during MA&R [45–47]. Thus, the objective of this study was to investigate the participants' experiences of the potential impact the MA&R had on their occupational engagement and to explore how the intervention's focus on occupations supported the participants' recovery process.

## 2. Material and Methods

### 2.1. Study Design

A qualitative study with a phenomenological-hermeneutic design [48–50] was chosen, to explore whether and how occupational engagement was affected through participation in MA&R, and if the occupation focused approach in MA&R, supported the participants' process of recovery. The phenomenological hermeneutic approach is a research method to elucidate and interpret peoples' meaning of their life worlds, situated in time and in everyday life. Guided by the theory of interpretation of Ricoeur, [51] a phenomenological-hermeneutic interpretation evolves over three steps: firstly, naive reading, structural analysis, and comprehensive understanding [48]. This study's point of departure was the understanding of the lived experiences of occupational engagement and personal recovery in relation to MA&R, as the phenomena was described by the participants. The study was conducted from December 2020 until May 2021, following the RCT intervention.

### 2.2. The MA&R Intervention

MA&R is based on principles from the Lifestyle Redesign ® program [52] and was developed into its current format in a collaboration between researchers, occupational therapists, and peer-workers employed in community mental health centres. The duration is approximately eight months and consists of 11 group-sessions and 11 one-on-one sessions led by an occupational therapist and a peer-worker (MA&R mentors). At group sessions, participants are introduced to topics related to meaningful activities and recovery, such as flow theory [53], storytelling, and strategies for occupational engagement, e.g. goalsetting. The MA&R mentors facilitate the sessions together, present themes, draw on examples from everyday life, and facilitate group exchange. The one-on-one sessions are held in conjunction with each group session and serve as a forum for further reflection on themes presented at the group sessions, to catch up with missing sessions, or to prepare for the following session. A detailed description of the MA&R is presented in the protocol paper by Bjørkedal et al. [44].

### 2.3. Participants and Settings

Thirteen participants were recruited from a larger sample of individuals with psychiatric disabilities, included in the MA&R RCT. MA&R was evaluated in a multicentre trial, with community mental health centres (CMCHs), a rehabilitation team, and activity and social support centres (ASSCs) as participating sites. The CMCHs delivered multidisciplinary treatment according to the Flexible-Assertive Community Treatment model, while the rehabilitation team delivered various rehabilitation services, mainly group based, such as self-esteem groups. The ASSCs were drop-in services, which means that they did not require referral or visitation. The ASSCs offered a wide range of activities, e.g., social happenings, open cafes, and creative activities. Participants in this study were affiliated to one of the sites when they enrolled in the MA&R trial.

The sampling strategy was based on maximal variation sampling regarding sites, sex, age, and time since completing the intervention, for variations in experiences to be explored [54, 55]. Participant selection criteria included men and women in various ages, recruited from the different sites (the rehabilitation team, ASSCs, and CMCHs) and those who had participated in MA&R in various timepoints before the interviews. We also aimed to include participants who had both completed and discontinued MA&R, but unfortunately, participants who have decided to discontinue MA&R either refused or did not respond to interview invitations. Sample size was deemed sufficient according to Malterud et al. That meant criteria for information power: study aim, sample specificity, use of established theory, quality of dialogue, and analysis strategy [56]. We found that our study aim was not broad, nor specific, but somewhat in between, as it encompassed occupational engagement and recovery (broad) in relation to the MA&R intervention (specific). The sample size was somewhat specific, as it entailed people with psychiatric disabilities who had been participating in MA&R. However, they were also a heterogenic group in terms of age, sex, life circumstances, type of psychiatric diagnosis, and recovery process. As the interviewer was an occupational therapist with work experiences within the population group, we expected the quality of dialogue to be adequate. The analysis strategy was informed by thematic analysis, search for cross-cases themes and nuances; hence, more participants are needed to be included than if we had deployed in-depth analysis. Based on these criteria we deemed that sample size should aim for about 12 to15 participants.

### 2.4. Data Collection

An interview guide was developed addressing the research question. Extracts from the interview guide are presented in Table 1. Semistructured interviews were conducted with a phenomenological approach using a narrative method to gain insights into the participants' experiences with MA&R, occupational engagement, and personal recovery. The interviews were conducted from December 2020 until February 2021. They were recorded digitally and transcribed verbatim and anonymized [49, 57]. Due to COVID19, personal interviews were limited, thus, nine of the interviews were conducted via videocall or cell phone, format was chosen by the informant and ranged from 45-75 minutes with a mean time of 62 minutes.

### 2.5. Analysis

The analysis strategy was guided by Malterud's Systematic text condensation (STC) [49, 58], a descriptive and explorative method inspired by phenomenology. The method involved the following steps: [1] reading all materials and obtaining an overall impression and bracketing previous preconceptions; then, reread with focus on the study aim; [2] identifying and sorting meaning units, representing different aspects of participants' experiences from their participation in MA&R, and coding; [3] condensing the contents and meanings of each of the coded groups; and [4] synthesizing the contents of each code group to generalize descriptions and concepts concerning engagement in activities and recovery.  Table 2 illustrates the analysis process. First and last author read the interview transcripts, discussed preliminary themes based on the overall impressions, identified and sorted meaning units, and developed codes. Contents and meaning where condensed and discussed, and finally synthesized by first, second, and last author.

### 2.6. Ethical Considerations

The study was conducted in conjunction to the MA&R RCT approved by the Danish Ethic Committee (H-18017307), and the Danish Data Protection Agency (VD-2018-299, I-Suite nr: 6543). It followed the principles from the Helsinki declaration [59]. Informants were informed about the study and its purpose and written informed consents were obtained. All references to individuals and quotations have been anonymized.

## 3. Results

### 3.1. Participants

Ten men and three women participated: age 25 to 50 years old. Four participants were students, the others were either job searching or received early retirement pension. The participants had various psychiatric diagnosis, about half had schizophrenia spectrum disorders. Participants had all completed MA&R, 0, 4, or 12 months prior to the interview (Table 3).

### 3.2. Findings

A hierarchical structure of themes was constructed during the inductive steps of analysis, revealing one overarching theme, capturing participants` overall perceptions of MA&R: *A practical approach to recovery*, along with three subthemes, each describing change processes in relation to occupational engagement and recovery (Figure 1).

#### 3.2.1. A Practical Approach to Recovery

MA&R was perceived as a pragmatic course, due to its future orientation towards activities and its nondiagnosis related curricula. Participants compared MA&R to having a personal trainer supporting engagement in activities. They valued the individual and flexible approach in MA&R and that they were free to engage in MA&R and in occupations, in their own pace, and according to their own offsets, for instance, not feeling that they should live up to explicit expectations about engaging in predefined activities. Participants highlighted this individually tailored approach as essential for their engagement. Some stated that they felt that there were major differences among them and the other persons participating in the group sessions. Not seeing common features or experiences among fellow group of participants impeded the participants feelings of connectedness and engagement during group sessions. Participants stated that the differences between them and other participants in the group, in respect to personal stages of recovery could be both a value and a hinder as those further along in these processes felt more alone.

“To me it was a little surreal, seeing that it was a recovery course, I expected it to be directed towards people who were a little more in the same state as me, where you have gone through the worst parts (illness red.) and is preparing to rebuild your everyday life—and there she (another participant) was in what seemed to be the worst crisis of her life—and here, by talking with my MA&R mentor, he enabled me to use less energy on other participants situation (…) where, in other group-settings I have become an “assistant-teacher” (…) and thus forgetting my own needs” (participant 4).

Here, the peer-worker enabled participants to draw parallels from the themes in MA&R and everyday life. Further, the peer-worker brought authenticity by still being in the recovery-process, introducing recovery as a possibility. Overall, participants perceived their engagement enhanced as they felt met with respect and equality from the MA&R mentors.

### 3.3. An Opportunity for Reorientation

#### 3.3.1. A Course, Not a Therapy

The fact that MA&R was a course and not a therapy was important to several of the participants before entering the course. It was valued that MA&R was not centred around illness or psychoeducation. Participants felt enabled to contemplate upon bettering their personal circumstances and valued the opportunity for personal exploration and perceptivity of everyday life.

“It was just what I could use, somebody who brings something positive and some ideas and suggestions, as to how I can better my life, without digging in what went wrong. And that is why I said “yes, please”, also because it was a course, not a therapy!” (participant 2).

Having the curricula in focus provided participants with a relaxed and informal climate during group sessions, where illnesses became less prominent. The focus on activities and recovery initiated a process of altering perspective. From going through the day on autopilot to identifying which activities they wanted to engage in, and thus discovering that they already had several meaningful activities in practice.

#### 3.3.2. I Will Take Advice from People Who See me

It was important for the individuals to feel recognized for their personality by MA&R mentors to perceive their encouragement as sincere. Hence engagement was fostered during the course when advice given was trusted e.g., MA&R mentors having a humble approach without dictating tasks. This inspired participants to engage enthusiastically throughout the course.

“One of the greatest things was their ability to see me. When the course ended, we all got a little postcard on how they perceived us and it was like they pointed out some things that weren't noticeable for me, and that was quite moving it made me feel very comfortable and there was a warmth to it, and it was not a clinical experience (…) but safe” (participant 9).

Feeling seen by the MA&R mentors, strengthened a sense of positive obligations in participants. Moreover, having the MA&R mentors to share their commitments with, promoted engagement in MA&R and a collaborative process around engaging in activities.

“It made me not give up, because hell, I wanted to be able to say that I did something, you know, when she (the OT) suggested something, then I had to try it out or try to look into it (..) it kept me on my feet, I had to do it before we saw each other again, whereas if it wasn't for the course, I would have been like “oh yeah, I will do it another day” and then it wouldn't amount to anything” (participant 13).

Conversely, not all participants did perceive MA&R as engaging. Some participants had entered MA&R with expectations of getting practical help or better managing everyday activities, so they became less arduous. They expressed disappointments by the end of the course, as they felt that these expectations were not met by the MA&R mentors, or they did not experience improvements in relation to performing everyday activities more effortless.

#### 3.3.3. It Is Right at my Grasp

It was commonly expressed that throughout MA&R, participants became aware that the term “activity” could be understood in several ways, in the sense that activities are individually defined as meaningful. Flow-theory and the discovery of absorption in seemingly mundane activities were highlighted by many as a concrete tool, easily available, and gradually adopted into ordinary day-to-day activities.

“It has definitely broadened my understanding of it (recovery), in the sense, that to me it is a rather uplifting thought, that it isn't just appointments with a psychologist or medication, that can stabilize me (…) but that these more concrete things, these small buttons, seemingly obvious buttons close to you, can mean that your symptoms can be dismantled” (participant 4).

Hereby, participants felt disburdened, enabling them to lower their expectations towards feelings of accomplishment now becoming more in line with their capabilities. It nurtured a curiosity of exploring meaning and pleasure in well-known everyday activities. The participants stated that it helped in applying a new perspective on daily activities available right at their grasp. However, one participant could not lower his expectations of authoring a book, for instance, by starting a process of write and rewrite, not aiming for the text to be perfect at first try, and felt inert, passive and not able to succeed during the course.

### 3.4. Meaning Making in Mundane Activities

#### 3.4.1. Small Things That Matter

Several participants stated that the “little things”, mundane, often taken-for-granted activities, were not irrelevant, just because they were “little”. They felt inspired by the idea of “size” of activities, “It's not either skydiving or sleeping, but it can be somewhere in between” (participant 7). Knowing that they need not do “grand” things, to make up a day of achievement, meant a greater appreciation towards ordinary elements in their everyday life. Several participants described that a new perspective led to further engagement in available tasks e.g., making plans to go shopping and engaging in self-care beforehand, now made grocery shopping a meaningful activity, or simply smiling or saying hello to a stranger there, meant having had an interaction that day.

“Just such a thing as watering the plant you haven't nurtured, after having starred at it for three weeks, hell, that quality of life. So, this has also changed. Definitely. In the sense that these smaller things they have a catalysing effect on many other things, like quality of life. And this is where I find meaning, in the small, close to home things” (participant 1).

Realizing that meaningful activities encompassed multiple types of activities that were deeply personal in terms of how they were performed and what meaning they had to people was highly valued among the participants. Identifying everyday activities that were meaningful, fostered self-determination in the participants, and helped them to avoid comparing themselves to others. Participants stated that this notion, made the meaningfulness more evident in the activities they were occupied with. It also enhanced their motivation to try out small activities, and their realization that not all practical tasks had to be chores but could also be enjoyable. Importantly, it was primarily these close to home activities that were possible. Social activities, such as seeking a tutor to initiate writing a book, or (re)establishing social relationships, were, for many participants, hindered by Covid-19 restrictions.

#### 3.4.2. Building a Basis

Some participants described that MA&R had altered their perceptions of their living situation, acknowledging its potential in rebuilding a steady fundament for wellbeing in everyday life. No longer a place to hide, the home became a safe environment and a catalyser for further activities. One participant who had a sleeping disorder as comorbidity, made her bedroom a sound space, since much of her time was spent there: adding flowers, making the bed, and airing out. Another participant let his spiritual beliefs stand out in his home, making it his sanctuary. Hence, meaningful engagement could be grounded in something as fundamental as watering ones plants.

“These meaningful activities are very close to home and daily life (….). It relates to taking care of myself, taking care of my home, and making this work, getting the basis to function” (participant 1).

One participant, however, did not feel satisfied as his wishes of wanting help to move and start over in a new place, could not be met by the MA&R mentors.

#### 3.4.3. I Am Not to Solve myself as a Problem

By focusing on existing resources, participants enhanced their awareness towards activities they already did, instead of focusing on the things they did not.

“…And realizing that everything doesn't have to be perfect according to other people's standards, but that you set your own standard, and the apartment does not have to be shiny and perfect. This is what I can do, this is my level, then other people can do what they are good at” (Participant 9).

Several participants described being more realistic about, and no longer ashamed of their capabilities. This led to a change of approach from neither-nor to “I can do both”, with limits. The acceptance fostered new insights, where disabilities were not a failure, but just a part of being that person at that time. This softened up a black and white perspective, where either you do the activity, or you do not. Participants experienced how formerly good activities felt detrimental when too much was initiated at once. This led to a focus upon what they could in fact do, creating more balance towards initiating activities in line with personal levels and meanings. Importantly, was to overcome the embarrassment that activities mundane to others, e.g., getting out of bed and on with the day, could be a struggle. Leading one participant with the courage to ask for help with his apartment, so that he could focus his energy upon engaging in other activities.

#### 3.4.4. My Toolbox of Resources

Throughout MA&R, participants felt supported in identifying their resources and utilizing these when engaging in activities, and conversely exploring how activities could be used as resources. Participants found it easier to engage in activities for their personal benefits, when they were curious about those in which they could fully immerse themselves. Participants reported that awareness and understanding of one's possibilities for wellbeing, when engaging in activity, came from realizing that focus was not devoted to symptoms if they were actively participating in activities. This gave rise to taking charge e.g., going to the park outside when sensing anxiety, or simply just placing yourself on the couch with a pet, just do something different. By noticing when activities felt good, opportunities arose to enforce these, and opposite, to distance from activities which felt draining.

Accessible activities became part of a personal toolbox. Walking became a proactive strategy for one participant when he felt apathic. Another started to take breaks to lean back and be attentive of own needs when his OCD took charge. Some participants focused on the feelings accompanied with an activity, such as tidying up could foster engagement and be enjoyable. Others adopted the notion that it is okay to slobber, when cleaning and not do 100%, which motivated to engage in activities.

“I have given myself permission to slobber, I like this principle of slobbering, at least now, so when I am cleaning, I do not have to get into every corner, but superficial cleaning is also a thing. Where before (…) when having to be this extreme, resulted in me not being able to handle anything at all” (participant 9).

### 3.5. On my Terms—A New Outlook on Everyday Life

#### 3.5.1. The Same, Yet an Altered Perspective

When asked about daily patterns and routines, most participants deemed that their everyday life looked the same as before MA&R, with few alterations. However, contemplation upon known routines and activities, stirred several participants away from “autopilot”, meaning that everyday life did not feel the same, due to an altered perspective of self-determination upon what makes up an activity.

“Tomorrow, we are going to the laundromat, and I am looking forward to it. The walk down there, and sometimes we sit and wait for the laundry to finish. And where this earlier was associated with a lot of anxiety, it has now become much better, to be able now to tell yourself “I'm just going to sit here”. But actually, being able to sit there, it gives me so much joy and all I want to do is improve this, what I have, more than I want to add anything, that's how I feel (Participant 9) ”.

Those participants who adopted new perspectives particularly did this in relation to “smaller” everyday activities, and by increasing their awareness of the opportunities these arose. For instance, one participant explained that bringing his camera, when taking a walk in the park, introduced new possibilities of experiencing a sense of flow when capturing nice motives. For some participants, routines were changed with emphasis upon favouring own needs and wants, e.g., one participant now started to make coffee as a morning routine:

“During my sick leave and while I was in MA&R, I practiced making myself a good cup of coffee every morning on my slow brewer, because making coffee or tea for myself was something I had never done, only if there were others” (Participant 4).

Reflecting on how activities could be a barometer for the recovery process, this participant reduced her working hours to resume good routines.

#### 3.5.2. Just Try It

MA&R created a space for trial and error where participants could experience success both inside and outside the group. Learning that engaging in activities took practice and not worrying about a “perfect outcome” was motivational and made it easier to initiate activities and feel more ease and presence in them.

“I would rather just try it out, and maybe it's not fun for me, or maybe I'm not good at it, but it might become enjoyable, or you could get better at it (…) but then you know your limits in that period and this might change as well” (participant 8).

One participant challenged his all-or-nothing approach, (job or no-job), and asked for job-training at the job centre, leading to developed job-abilities, slowly easing his way back to work-life routines.

This contributed to a different approach to activities, as opportunities for creating momentums.

“I think there is a positive spill over effect, if something is enjoyable, then it becomes easier to do other things too” (Participant 11).

#### 3.5.3. I Can Feel Good about What I Do

Some participants expressed being able to, to some degree, manage their own wellbeing through activities. Participants highlighted that learning about flow-theory and being able to identify with a state of flow, was a positive experience. Knowing that flow could appear in their natural environment merely by putting on music or folding laundry, made participants aware that this was attainable for them and that they could feel “normal”.

“I have become aware of it (flow red.), and I think that is the important part. I have become aware that I, for brief periods can feel like everybody else and be occupied by something and go into that state. That process is what has become clear to me” (Participant 1).

Initially, it required a lot of awareness to engage, but over time “just” engaging in activities became more intuitive e.g., by taking your camera with you on a walk. By focusing on “the good” in activities and letting achievements outweigh defeats, several participants were enabled to see possibilities in their surroundings, where the “to-do” list was replaced with a “try-this” list. When a participant in the interview was asked if she was better able to do what she wanted to do, she answered:

“Yes, I feel that I am, that I do. There is always that thought when you deal with recurring mental illness “it will come back”, you know? Right now, I am on a positive road, and hopefully, when it goes uphill again, then I will try and focus more on doing some of the things that I have discovered makes me happy and does me good, by taking me out of my head—having had this year to figure out what these things were” (Participant 13).

The participants felt more equipped to verbalize their concerns and avoid situations that could result in defeat. Several participants felt more able to express their needs towards friends and family.

#### 3.5.4. Moving on to an Open World

Through engagement in activities and by enhancing the experiences of respite, participants felt their illness less prominent. This made recovery seem attainable by using activities as an indicator for mental wellbeing, e.g., the reattainment of bicycling or the awareness of skipping good morning routines.

“I remember how good it felt when I started riding my bicycle around town again, because I have always identified myself as one of those city-types who rides their bicycle around town. But all those years being ill I only took the bus, and I was in the back of the bus hiding, primarily riding the bus in knowing, that in this place I wouldn't run in to anybody I knew. (…), and it made a huge difference for me when I started bicycling again, because it was a recognition that, all right, now I am aware that I can possibly run into someone, so in doing this I felt like I moved on to an open world again” (Participant 4).

Choosing daily activities more in tune with own preferences such as their ability of feeling absorbed or respite or simply perceiving taking a break as an activity, nurtured hope, and experience of living meaningful lives. Several participants also spoke of the possibility of becoming peer-workers themselves.

## 4. Discussion

The findings in this study illuminate whether and how MA&R supported activity engagement and subsequently, the recovery process from the participants' perspectives. The program's emphasis on reorientation in daily life, for instance in relation to meaning making of occupational experiences, and rethinking interests, values, aspirations, and identities, the personal orientation, and its pragmatic approach with emphasis on trial and error was highlighted by the participants. The activity-oriented focus, together with a respectful tone, supported participants to engage and experience meaning in activities within their reach during MA&R. Participants adopted several considerations for mundane activities learning that these could provide joy and immersion, and their homes and surrounding became pivotal for wellbeing and a safe space to recoup.

### 4.1. Occupational Engagement and Recovery

Our findings align with results from Sommer et al.'s metasynthesis on recovery [60], identifying three key processes: being, doing, and accessing. Contextualized by the constraints psychiatric disabilities encompass, these processes' make everyday life experiences into opportunities for accessing resources, enjoyments, and new possibilities intertwined with opportunities for recovery. In their metasynthesis [60] being and doing are described as generic recovery processes. *Being* refers to the temporal unfolding of meaning, being well in everyday life, belonging, and accepting. *Doing* refers to participating and contributing through everyday activities within a social context where the person feels valued. In our study, participants distinguished between daily life looking the same, and feeling the same. We interpret this as recovery through the descriptions from MA&R participants, possibly being closely linked to temporality and occupational engagement, more than to occupational performance. This poses a question whether MA&R first and foremost support recovery in terms of wellbeing and experiences of meaning, and how this can be achieved with or without making actual changes in daily activities, but by changing perspective. Contemplating on the findings, that the smaller day-to-day activities took presence could be a result of the Covid19 pandemic, having affected *accessing*—the third process by Sommer et al., when restrictions and lockdowns closing opportunities to attend activities in the greater social surroundings. Thus, restrictions could have had serious consequences on quality of life [61–64]. But, having had an altered perspective on daily routines and quality of life, participants perhaps saw possibilities ahead and felt that everyday life was more in tune with wishes, which depicts having more attention towards building a solid basis where one could feel good. By change of perspective, making changes in day-to-day activities, otherwise not clear, become noticeable.

Present results also have ties to findings from a scoping review by Doroud et al. [16], examining recovery seen through occupational engagement, discovering a process set in three interrelated stages with impact on personal recovery (CHIME) [20]. Standing out in the current study are especially the first two processes: (i) recovery as gradual occupational reengagement—doing to get started and (ii) recovery as engaging within the stream of everyday occupational life. The latter, (iii) recovery as full community participation and citizenship, was partly disrupted by the pandemic.

Activities on hand and their tangibility through trials rendered as a solid basis, and a prominent theme appeared through the interviews, that daily life did not feel the same by applying a new focus of temporality whilst being in activity. By working with “trial and error” in activities in- and outside MA&R, engaging in these became less fearful through the perception of it as practice for the “real world”. This is in line with Doroud et al. [16], who found that small tasks can help a person rediscover hope and constructively reappraise their capabilities and resources. Several participants expressed that accepting one's own capabilities was difficult but was aided in the individual meetings with MA&R mentors, helping decrease demands towards oneself, accommodating them to set their own standard for meaningful activities. Hereby, in line with other research from Black and colleagues [15], *a subjective experience of engagement* became clear, with examples such as riding the bicycle across town again, being mindful about the bedroom or the different aspects of going to the laundromat, and just *be* with a friend.

Although there often might be overlaps between activities that are culturally and personally valued (e.g. work is a social expectation in most cultures, and at the same time personally significant to people) [65, 66], findings in this study suggest that meaning making in activities are, when narrowed down, *in the eye of the beholder.* People have different ideas about what make meaning in their lives. Consequently, promoting occupational engagement is not a process that should be taken for granted by merely assuming what kind of occupational opportunities people with psychiatric disabilities need, for instance by building mental health services that solely offer predefined activities. Assisting a person to discover where feelings of absorption appear, and to strengthen the awareness of activities, mundane, familiar, or new, can foster a feeling of connectedness to everyday life. Enabling the person to build upon the personally defined occupational life, in line with Doroud et al. [16] can support *recovery through engagement in the stream of everyday life.*

Findings from this study stress the importance of meeting the person's recovery goals. Participants became disengaged when they did not feel met by the MA&R mentors. Persson et al. proposes in their analysis of value dimensions, meaning and complexity in occupations, that occupations have symbolic value on a personal and cultural level. Through choices of occupations, the individuals communicate aspects of themselves, to the immediate world. The social environment communicates “back”, to the doer, providing feedback on whether the behaviour is acceptable and valuable according to cultural norms and ideologies. [67] Participants who felt met, seen, and/or supported in MA&R, began a process of putting less emphasis on the symbolic value in occupations from a cultural level. Participants described being less ashamed of not being able to perform activities taken for granted by broader society, such as getting up and on with the day. They also stated that MA&R helped them avoid comparing themselves to others. Instead, MA&R supported an exploration of the symbolic value in occupations on a personal level, acknowledging that lying on the couch with a pet, or taking photos in the park, where significant activities if they mattered to the participants. This shift of focus might for some participants have led to a greater self-acceptance and soften up a critical self-image of a person having disabilities. Towards putting more emphasis on the symbolic value in occupations on a personal level. This may have fostered gradual occupational reengagement [16] and initiating a positive cycle to experiment further in other activities, because of their potential of enjoyment, FLOW, or sense of accomplishment. It may also have aided participants to *develop identity through occupation* [15] in knowing their limits and gaining a stronger sense of self, which is needed to withstand the effects of negative expectations and stereotyping from the broader community [68].

Findings from this study point to both similarities and differences with qualitative studies on participants experiences with BEL [35–37], AOI [38], and OMP [34]. Perceiving MA&R as a practical take on recovery aligns with results from studies investigating participants experiences in relations to AOI and OMP. Findings from these studies showed that reflecting on the meaning in occupations and acknowledging the links between occupations, health, and wellbeing, facilitated feelings of hope and agency, and a sense of normality [34, 38]. Similar to participants from the OMP [34] study and the BEL study [36], participants in MA&R described developing confidence, which enabled them to dare to try out or reengage in activities that mattered to them. The programs resolving on the meaning and value of small, mundane activities seemed highly valued among participants, and indicate that providing people with psychiatric disabilities knowledge and opportunities to explore and engage in occupations might create new pathways to recovery by strengthening a positive identity, providing new sources of meaning, building connectedness, nurturing hope, and empowerment [34–36, 38]. One striking difference between the findings in MA&R, and the results from the BEL, OPM, and AOI study was that the participants did not perceive peer-support among group participants as a supportive element in the intervention. They found that perceived differences between themselves and the other participants in the group was a barrier for engagement. Instead, participants in MA&R highlighted the peer-workers' role, for showing them new opportunities for engagement, and for drawing parallels between the sessions and their everyday lives. Thus, having occupational therapist and a peer-worker codelivering sessions make good sense to the participants, and may strengthen the program's potential impacts. Coproductions between peer-workers and occupational therapists, when developing occupation focused program, should also be considered when developing and refining recovery-oriented interventions targeting occupational engagement. Also, the individual approach in MA&R, was highly valued, which indicate that adding one-on-one sessions to group-based interventions may be a useful tool for tailoring person-oriented services. Participants' notion of feeling seen by the MA&R mentors was more prominent in the MA&R study, than in BEL [35, 37], AOI [38], and OPM [34], which suggest that combining individual sessions and support with group sessions, might foster distinct change processes in relation to occupational engagement. However, this needs further explorations. Overall, the findings in this study suggest that MA&R can be a relevant recovery-oriented approach as it addresses occupational engagement, an important recovery goal for people with mental illness. The MA&R RCT was a multicentre trial, and the program was delivered in both municipality mental health services and in community mental health centres, which indicate that the MA&R format may fit into various mental health settings were occupational therapists and peer-workers are employed.

### 4.2. Methodological Considerations

A stepwise purposeful sampling [54] was chosen within this somewhat homogeneous group of participants, seeking variation within different timepoints since enrolment in MA&R. Albeit, we were not able to sufficiently recruit in relation to demographic criteria, as male participants dominated, thus addition of female participants would have been advantageous. Due to COVID19, personal interviews were limited, thus nine of the interviews were conducted via telephone or videocall, the remaining four participants emphasized face-to-face interviews, leading to variations of data collection. The first author carefully secured a safe space to express thoughts invariably, and quality was not deemed affected by this fact.

While phenomenological philosophy is not as explicitly stated in STC as in Giorgi's method [69] or Interpretative Phenomenological Analysis [70], STC still shares the foundations of life-world experiences as valid knowledge [58]. STC in the current study procedure was invoked as a committed phenomenological analysis, a strategy chosen to bring forth the essence of the phenomenon [49, 58, 71]. During all steps of the research process a commitment to reflexivity was held [49, 71–73]. Early in the process, preconceptions were identified and returned to during analysis to secure bracketing. This was done by first author, who kept a reflexive journal during the research process, and wrote memos after interviews, and by last author who wrote down assumptions about participants' experiences with MA&R, prior to initiating the study [73].

To enhance trustworthiness and improve credibility, authors were engaged in a constant dialogue to consolidate on each level in the analysis, thus supplementing and contesting each other's findings to strengthen the understanding of the phenomena [71, 74, 75]. STC also explicitly prescribes recontextualization as the final step of analysis, validating interpretations and findings against the initial complete transcripts. However, the authors conducting the analysis were all trained occupational therapists, which may increase the risk of blind angles while consolidating the themes and interpretating the findings [49].

## 5. Conclusion and Clinical Implications

Findings from this study show that MA&R was perceived as a practical approach to recovery and that the activity focus in MA&R supported this approach. Participants highlighted the experiences of recovery through the “small things” in life, often taken for granted. They appreciated MA&R for its positive and future-orientation and personalized approach alongside opportunities for trial and error. The findings provided understandings of how occupational engagement and recovery are intertwined and manifested through everyday experiences. Aiding in personal recovery was an altered perspective upon activities, challenging the “big” or “small” activities and applying own terms towards meaningfulness and presence in daily life. Moreover, the findings indicate that occupational engagement can be enhanced, with or without increased occupational performance.

The MA&R course-setup enabled participants motivation to take-in curricula and apply knowledge towards activities. Knowledge was empowering in giving participants tools right at their grasp. The results from our study suggest that MA&R supported the participants in developing a new “lens” on meaningful activities—highlighting the value of everyday experiences for recovery and wellbeing.

## Figures and Tables

**Figure 1:** Overview of themes: Overarching theme, main themes, and subthemes.

**Table 1:** Extract from interview guide.

Research question	Examples of questions posed in the interview
Whether and how MA&R enabled activity engagement is seen from the participants perspectives	How would you describe MA&R to me, assuming I had never heard of it? If/how did the course affected your view or reflection upon activities in your daily life? Have you explored new aspects of your daily life since entering the course?
Whether and how the intervention's embedded focus on activities supported the participants' recovery process	Has the course provided you with activities? Has participation in the course enabled you to do more of what you want? Has participation in the course changed the way you think about quality of life?

**Table 2:** Illustration of the analysis process from meaning unit to theme.

Citation number	Meaning unit	Condensed	Code group	Theme
194	“And were I saw no possibility for attaining any sort of recovery or getting any sort of meaningful activities into my daily life, I do have a positive view on this today, and that is partly because I dared to ask for help, because this entails a great deal of embarrassment to me. I find it embarrassing to ask for help for things that other people do not even think about, but just do. Or at least that is what I tell myself”	Taking initiative and asking for help to attain my apartment, made me look positive on recovery as a possibility for me. Daring to face the perceived embarrassment was a big step.	Abilities: Taking charge asked for help. Respite	I am not to solve myself as a problem.
195	“You know what, maybe it just has not sunken in yet, because that's right, taking the initiative to ask for help that is a big deal, that is a very big deal. So yes of course, something has happened within me and as I said, asking for this help, help with my apartment, is a result of this project”			

**Table 3:** Description of participants.

Participant number and gender	Age/range	Diagnosis	Employment status	Time since MA&R
(1) Male	40-45	Schizophrenia	Early retirement	4 months
(2) Female	45-50	Attention deficit hyperactive disorder, borderline personality disorder, and PTSD	Early retirement	One year
(3) Male	25-30	Schizophrenia	Welfare	One year
(4) Female	30-35	Depression	Job training	2 months
(5) Male	50-55	Depression	Job	4 months
(6) Male	20-25	Obsessive compulsive disorder, generalized anxiety, and stress	Student	Finishing
(7) Male	50-55	Unknown	Early retirement	Finishing
(8) Male	25-30	Schizotypal personality disorder	Student and job seeking	4 months
(9) Male	35-40	Schizotypal personality disorder	Job seeking	One year
(10) Male	45-50	Obsessive compulsive disorder	Early retirement	Finishing
(11) Male	30-35	Schizophrenia	Student and job seeking	Finishing
(12) Male	30-35	Psychosis and stress	Student	Finishing
(13) Female	45-50	Depression	Early retirement	3 months

## Data Availability

The datasets used and/or analysed during the current study are not available, due to Danish Law and GPDR.
